RETRACTED

# Oxonium picrate

**DOI:** 10.1107/S1600536811022574

**Published:** 2011-06-18

**Authors:** Shou-Wen Jin, Bing-Xia Chen, Yu-Shuang Ge, Hua-Bing Yin, Yu-Ping Fang

**Affiliations:** a Tianmu College, ZheJiang A & F University, Lin’An 311300, People’s Republic of China

## Abstract

The title compound, H_3_O^+^·C_6_H_2_N_3_O_7_^−^, consists of one picrate anion and one oxonium cation. The oxonium cation is located on a crystallographic twofold axis and both its H atoms are disordered, each over two symmetry-equivalent positions with occupancy ratios of 0.75. The picrate anions are also located on twofold axes bis­ecting the phenolate and *p*-nitro groups. π–π inter­actions between the rings of the picrates [centroid-to-centroid distances of 3.324 (2) Å] connect the anions to form stacks along the *a*-axis direction. The stacks are further joined together by the protonated water mol­ecules through hydrogen bonds to form two-dimensional sheets extending parallel to the *ab* plane. The sheets are stacked on top of each other along the *c*-axis direction and connected through C—H⋯O inter­actions between the CH groups of the benzene rings and the picrate nitro groups, with C⋯O distances of 3.450 (2) Å.

## Related literature

For general background to organic salts of picric acid, see Jin *et al.* (2010 ▶); Harrison *et al.* (2007 ▶); Muthamizhchelvan *et al.* (2005 ▶); Smith *et al.* (2004 ▶).

## Experimental

### 

#### Crystal data

H_3_O^+^·C_6_H_2_N_3_O_7_^−^
*M* *_r_* = 247.13
Orthorhombic,
*a* = 7.1510 (6) Å
*b* = 19.80820 (18) Å
*c* = 13.50610 (12) Å
*V* = 1913.12 (16) Å^3^
*Z* = 8
Mo *K*α radiation
μ = 0.16 mm^−1^
*T* = 298 K
0.45 × 0.34 × 0.31 mm

#### Data collection

Bruker SMART CCD area-detector diffractometer
Absorption correction: multi-scan (*SADABS*; Bruker, 2002 ▶) *T*_min_ = 0.936, *T*_max_ = 0.951
3842 measured reflections
848 independent reflections
654 reflections with *I* > 2σ(*I*)
*R*_int_ = 0.044

#### Refinement

*R*[*F* ^2^ > 2σ(*F* ^2^)] = 0.044
*wR*(*F* ^2^) = 0.140
*S* = 1.12
848 reflections
89 parameters
2 restraints
H atoms treated by a mixture of independent and constrained refinement
Δρ_max_ = 0.21 e Å^−3^
Δρ_min_ = −0.41 e Å^−3^

### 

Data collection: *SMART* (Bruker, 2002 ▶); cell refinement: *SAINT* (Bruker, 2002 ▶); data reduction: *SAINT*; program(s) used to solve structure: *SHELXS97* (Sheldrick, 2008 ▶); program(s) used to refine structure: *SHELXL97* (Sheldrick, 2008 ▶); molecular graphics: *SHELXTL* (Sheldrick, 2008 ▶); software used to prepare material for publication: *SHELXTL*.

## Supplementary Material

Crystal structure: contains datablock(s) global, I. DOI: 10.1107/S1600536811022574/zl2375sup1.cif

Structure factors: contains datablock(s) I. DOI: 10.1107/S1600536811022574/zl2375Isup2.hkl

Supplementary material file. DOI: 10.1107/S1600536811022574/zl2375Isup3.cml

Additional supplementary materials:  crystallographic information; 3D view; checkCIF report

RETRACTED

## Figures and Tables

**Table 1:** Hydrogen-bond geometry (Å, °)

*D*—H⋯*A*	*D*—H	H⋯*A*	*D*⋯*A*	*D*—H⋯*A*
O5—H5*B*⋯O2^i^	0.91 (2)	2.17 (2)	3.061 (3)	166 (5)
O5—H5*A*⋯O1	0.92 (2)	1.93 (2)	2.848 (2)	172 (5)
C3—H3⋯O3^ii^	0.93	2.52	3.450 (2)	175

Symmetry codes: (i) ; (ii) .

## supplementary crystallographic information

### Comment

It is well known that picric acid is used primarily to prepare explosives, and as an intermediate to manufacture dyes. As a strong organic acid, picric acid forms salts with many N-containing organic bases (Smith *et al.*, 2004; Harrison *et al.*, 2007; Muthamizhchelvan *et al.*, 2005). As an extension of our study concerning organic salts based on picric acid (Jin *et al.*, 2010), we herein report the crystal structure of oxonium picrate.

The single crystal of the title compound (Fig. 1) with the formula C_6_H_5_N_3_O_8_ was obtained by recrystallization of picric acid and 2-chloropyridine from a methanol solution. However the 2-chloropyridine molecules do not appear in the title compound. X-ray diffraction analysis indicated that in the title compound there are one protonated water molecule, and one picrate. The OH group of the picric acid is ionized and the proton is transferred to the water molecule. In the title compound all of the bond distances and angles are in the normal range. The oxonium cation is located on a crystallographic two-fold axis and both its H atoms are disordered over each two symmetry equivalent positions with occupancy rates of 0.75 each. The benzene ring of the picrate is almost planar. The *ortho*-nitro groups (N1—O2—O3, and N1A—O2A—O3A) deviate from the benzene ring plane and have a dihedral angle of 25.6 (2)° with the benzene plane, whereas the *para*-nitro group lies almost in the benzene plane [with a dihedral angle of 2.0 (1)° between the N2—O4—O4A group and the benzene ring]. These structural data are similar to those in other structurally described picrates (Muthamizhchelvan *et al.*, 2005).

π–π Interactions between the phenyl rings of the picrates (with Cg–Cg distances of 3.324 (2) Å) connect the picrate anions to form stacks along the a axis direction. Within one stack molecules alternate and are arranged in an antiparallel fashion. The one-dimensional picrate stacks are further linked together by the oxonium ions to form a two-dimensional sheet structure when it is viewed from the *c* axis direction (Fig. 2). The sheets are further stacked along the *c* axis direction through CH—O interactions between CH of the benzene rings and the nitro groups of the picrates with C—O distances of 3.450 (2) Å to form a three-dimensional structure.

RETRACTED

### Experimental

Crystals of oxonium picrate were formed by slow evaporation of its methanol solution at room temperature. Picric acid (23 mg, 0.10 mmol) was dissolved in 4 ml of methanol, and 2-chloropyridine (11 mg, 0.10 mmol) was added to the methanol solution. The solution was then filtered into a test tube and left standing at room temperature. After about one week yellow block crystals were obtained.

### Refinement

H atoms H5A and H5B bonded to the oxonium O atom were located in a difference Fourier map and refined isotropically. The oxonium cation is located on a crystallographic two-fold axis and both H5A and H5B are disordered over each two symmetry equivalent positions, and both have an occupancy of 0.75. Other H atoms were positioned geometrically with C—H = 0.93 Å for aromatic H atoms, and constrained to ride on their parent atoms with *U*_iso_(H) = 1.2U_eq_(C).

### Crystal data

**Table:**

H_3_O^+^·C_6_H_2_N_3_O_7_^−^	*D*_x_ = 1.716 Mg m^−^^3^
*M**_r_* = 247.13	Mo *K*α radiation, λ = 0.71073 Å
Orthorhombic, *I**b**c**a*	Cell parameters from 1867 reflections
*a* = 7.1510 (6) Å	θ = 1.5–25.0°
*b* = 19.80820 (18) Å	µ = 0.16 mm^−^^1^
*c* = 13.50610 (12) Å	*T* = 298 K
*V* = 1913.12 (16) Å^3^	Block, yellow
*Z* = 8	0.45 × 0.34 × 0.31 mm
*F*(000) = 1008	

### Data collection

**Table:**

Bruker SMART CCD area-detector diffractometer	848 independent reflections
Radiation source: fine-focus sealed tube	654 reflections with *I* > 2σ(*I*)
graphite	*R*_int_ = 0.044
φ and ω scans	θ_max_ = 25.0°, θ_min_ = 2.1°
Absorption correction: multi-scan (*SADABS*; Bruker, 2002)	*h* = −8→8
*T*_min_ = 0.936, *T*_max_ = 0.951	*k* = −22→23
3842 measured reflections	*l* = −16→6

### Refinement

**Table:**

Refinement on *F*^2^	Secondary atom site location: difference Fourier map
Least-squares matrix: full	Hydrogen site location: inferred from neighbouring sites
*R*[*F*^2^ > 2σ(*F*^2^)] = 0.044	H atoms treated by a mixture of independent and constrained refinement
*wR*(*F*^2^) = 0.140	*w* = 1/[σ^2^(*F*_o_^2^) + (0.0677*P*)^2^ + 3.1011*P*] where *P* = (*F*_o_^2^ + 2*F*_c_^2^)/3
*S* = 1.12	(Δ/σ)_max_ < 0.001
848 reflections	Δρ_max_ = 0.21 e Å^−^^3^
89 parameters	Δρ_min_ = −0.41 e Å^−^^3^
2 restraints	Extinction correction: *SHELXL97* (Sheldrick, 2008), Fc^*^=kFc[1+0.001xFc^2^λ^3^/sin(2θ)]^-1/4^
Primary atom site location: structure-invariant direct methods	Extinction coefficient: 0.039 (4)

### Special details

**Table:**

Geometry. All e.s.d.'s (except the e.s.d. in the dihedral angle between two l.s. planes) are estimated using the full covariance matrix. The cell e.s.d.'s are taken into account individually in the estimation of e.s.d.'s in distances, angles and torsion angles; correlations between e.s.d.'s in cell parameters are only used when they are defined by crystal symmetry. An approximate (isotropic) treatment of cell e.s.d.'s is used for estimating e.s.d.'s involving l.s. planes.
Refinement. Refinement of *F*^2^ against ALL reflections. The weighted *R*-factor *wR* and goodness of fit *S* are based on *F*^2^, conventional *R*-factors *R* are based on *F*, with *F* set to zero for negative *F*^2^. The threshold expression of *F*^2^ > σ(*F*^2^) is used only for calculating *R*-factors(gt) *etc*. and is not relevant to the choice of reflections for refinement. *R*-factors based on *F*^2^ are statistically about twice as large as those based on *F*, and *R*-factors based on ALL data will be even larger.

RETRACTED

### Fractional atomic coordinates and isotropic or equivalent isotropic displacement parameters (Å^2^)

**Table:**

	*x*	*y*	*z*	*U*_iso_*/*U*_eq_	Occ. (<1)
N1	0.3838 (3)	0.11353 (11)	0.17214 (16)	0.0328 (7)	
N2	0.2500	−0.09568 (15)	0.0000	0.0361 (8)	
O1	0.2500	0.18513 (12)	0.0000	0.0369 (8)	
O2	0.3327 (3)	0.17048 (10)	0.19325 (15)	0.0502 (7)	
O3	0.4947 (3)	0.08131 (11)	0.22328 (15)	0.0497 (7)	
O4	0.3100 (4)	−0.12491 (10)	0.07276 (19)	0.0630 (8)	
O5	0.0000	0.2500	0.1338 (2)	0.0489 (9)	
H5A	0.089 (6)	0.233 (3)	0.091 (3)	0.073*	0.75
H5B	0.052 (7)	0.279 (2)	0.177 (3)	0.073*	0.75
C1	0.2500	0.12179 (17)	0.0000	0.0270 (8)	
C2	0.3107 (4)	0.08102 (13)	0.08289 (17)	0.0270 (7)	
C3	0.3134 (4)	0.01147 (13)	0.08305 (17)	0.0286 (7)	
H3	0.3569	−0.0122	0.1378	0.034*	
C4	0.2500	−0.02233 (17)	0.0000	0.0282 (8)	

### Atomic displacement parameters (Å^2^)

**Table:**

	*U*^11^	*U*^22^	*U*^33^	*U*^12^	*U*^13^	*U*^23^
N1	0.0376 (14)	0.0358 (13)	0.0250 (12)	−0.0067 (10)	−0.0014 (10)	0.0001 (9)
N2	0.0350 (19)	0.0269 (16)	0.046 (2)	0.000	0.0059 (15)	0.000
O1	0.0587 (19)	0.0226 (13)	0.0295 (14)	0.000	0.0085 (13)	0.000
O2	0.0748 (17)	0.0372 (12)	0.0387 (12)	0.0047 (10)	−0.0128 (11)	−0.0126 (9)
O3	0.0569 (15)	0.0538 (13)	0.0385 (12)	0.0006 (11)	−0.0193 (10)	0.0019 (9)
O4	0.096 (2)	0.0300 (12)	0.0629 (15)	0.0117 (11)	−0.0140 (14)	0.0089 (10)
O5	0.061 (2)	0.0414 (17)	0.0443 (18)	−0.0008 (15)	0.000	0.000
C1	0.0273 (19)	0.0275 (18)	0.0260 (18)	0.000	0.0050 (14)	0.000
C2	0.0287 (14)	0.0305 (14)	0.0217 (13)	−0.0032 (10)	0.0009 (10)	−0.0014 (9)
C3	0.0279 (14)	0.0303 (14)	0.0275 (13)	0.0010 (11)	−0.0001 (11)	0.0051 (10)
C4	0.0262 (19)	0.0248 (17)	0.0337 (19)	0.000	0.0041 (15)	0.000

### Geometric parameters (Å, °)

**Table:**

N1—O2	1.220 (3)	O5—H5B	0.91 (2)
N1—O3	1.230 (3)	C1—C2	1.447 (3)
N1—C2	1.463 (3)	C1—C2^i^	1.447 (3)
N2—O4	1.219 (3)	C2—C3	1.378 (4)
N2—O4^i^	1.219 (3)	C3—C4	1.383 (3)
N2—C4	1.453 (5)	C3—H3	0.9300
O1—C1	1.255 (4)	C4—C3^i^	1.383 (3)
O5—H5A	0.92 (2)		
			
O2—N1—O3	122.8 (2)	C3—C2—C1	124.3 (2)
O2—N1—C2	119.5 (2)	C3—C2—N1	115.7 (2)
O3—N1—C2	117.7 (2)	C1—C2—N1	119.9 (2)
O4—N2—O4^i^	123.3 (3)	C2—C3—C4	118.6 (2)
O4—N2—C4	118.37 (17)	C2—C3—H3	120.7
O4^i^—N2—C4	118.37 (17)	C4—C3—H3	120.7
H5A—O5—H5B	111 (5)	C3^i^—C4—C3	122.1 (3)
O1—C1—C2	123.92 (15)	C3^i^—C4—N2	118.97 (16)
O1—C1—C2^i^	123.92 (15)	C3—C4—N2	118.97 (16)
C2—C1—C2^i^	112.2 (3)		
			
O1—C1—C2—C3	−179.13 (18)	C1—C2—C3—C4	−1.7 (3)
C2^i^—C1—C2—C3	0.87 (18)	N1—C2—C3—C4	−178.59 (19)
O1—C1—C2—N1	−2.4 (3)	C2—C3—C4—C3^i^	0.81 (17)
C2^i^—C1—C2—N1	177.6 (3)	C2—C3—C4—N2	−179.19 (17)
O2—N1—C2—C3	−155.8 (3)	O4—N2—C4—C3^i^	178.42 (19)
O3—N1—C2—C3	23.8 (3)	O4^i^—N2—C4—C3^i^	−1.58 (19)
O2—N1—C2—C1	27.2 (3)	O4—N2—C4—C3	−1.58 (19)
O3—N1—C2—C1	−153.3 (2)	O4^i^—N2—C4—C3	178.42 (19)

Symmetry codes: (i) −*x*+1/2, *y*, −*z*.

RETRACTED

### Hydrogen-bond geometry (Å, °)

**Table:**

*D*—H···*A*	*D*—H	H···*A*	*D*···*A*	*D*—H···*A*
O5—H5B···O2^ii^	0.91 (2)	2.17 (2)	3.061 (3)	166 (5)
O5—H5A···O1	0.92 (2)	1.93 (2)	2.848 (2)	172 (5)
C3—H3···O3^iii^	0.93	2.52	3.450 (2)	175

Symmetry codes: (ii) −*x*+1/2, −*y*+1/2, −*z*+1/2; (iii) *x*, −*y*, −*z*+1/2.

## References

[bb1] Bruker (2002). *SADABS*, *SMART* and *SAINT* Bruker AXS Inc., Madison, Wisconsin, USA.

[bb2] Harrison, W. T. A., Swamy, M. T., Nagaraja, P., Yathirajan, H. S. & Narayana, B. (2007). *Acta Cryst.* E**63**, o3892.

[bb3] Jin, S. W., Zhang, W. B., Liu, L., Gao, H. F., Wang, D. Q., Chen, R. P. & Xu, X. L. (2010). *J. Mol. Struct.* **975**, 128–136.

[bb4] Muthamizhchelvan, C., Saminathan, K., Fraanje, J., Peschar, R. & Sivakamar, K. (2005). *Anal. Sci.* **21**, x61–x62.

[bb5] Sheldrick, G. M. (2008). *Acta Cryst.* A**64**, 112–122.10.1107/S010876730704393018156677

[bb6] Smith, G., Wermuth, U. D. & Healy, P. C. (2004). *Acta Cryst.* E**60**, o1800–o1803.10.1107/S010827010401505715295198

